The article "The Effects of Acute Caffeine Supplementation on Performance in Trained CrossFit Athletes" was retracted in 2020. Reasons: errors in the analysis; errors in the methods; errors in the results or conclusions.

# The Effects of Acute Caffeine Supplementation on Performance in Trained CrossFit Athletes

**DOI:** 10.3390/sports7040095

**Published:** 2019-04-25

**Authors:** Jesse A. Stein, Melitza Ramirez, Katie M. Heinrich

**Affiliations:** Department of Kinesiology, College of Human Ecology, Kansas State University, Manhattan, KS 66506, USA; melitzar@ksu.edu (M.R.); kmhphd@ksu.edu (K.M.H.)

**Keywords:** high intensity functional training, exercise, males, muscular endurance, ergogenic aids, sports nutrition

## Abstract

Caffeine’s ergogenic effects persist during various exercise modalities; however, information establishing its efficacy during CrossFit protocols is limited. Our study aimed to determine the effects of caffeine supplementation on CrossFit performance. Thirteen CrossFit-trained men (age = 28.5 ± 6.6 years, experience = 49.2 ± 36.3 months) were randomized in a double-blind, crossover design. Participants completed two sessions separated by a seven-day washout period, 60 min after consuming 5 mg/kg body mass of caffeine or a placebo. In each session, participants completed as many rounds as possible in 20 min of 5 pull-ups, 10 push-ups, and 15 air squats. CrossFit performance was the total number of repetitions completed in 20 min. Paired samples t-tests were used to compare CrossFit performance between caffeine and placebo conditions and to test for a potential learning effect between the first and second sessions. CrossFit performance was significantly higher during the caffeine condition compared to the placebo (461.4 ± 103 vs. 425.0 ± 93.5 repetitions, *p* < 0.05). No significant learning effect was identified between the first and second sessions (445.6 ± 95.0 vs. 440.8 ± 105.0 repetitions, *p* = 0.73) nor was there a significant treatment order effect (*p* = 0.40). Caffeine’s ergogenic effect is present during CrossFit; however, future investigations should establish caffeine’s efficacy during other CrossFit protocols and among female athletes.

## 1. Introduction

Caffeine supplementation is pervasive in sporting disciplines with 74% of elite athletes consuming caffeine prior to competition for its ergogenic effects [1]. Support for this strategy is recognized by the International Olympic Committee and the International Society of Sports Nutrition who both acknowledge caffeine as a dietary supplement with ‘good evidence’ for its ergogenic effects, benefiting endurance and strength/power in athletes [2,3,4,5]. A majority of this evidence has been established utilizing singular exercise modalities when assessing muscle function (muscular strength and endurance) or exhaustive protocols (time-to-exhaustion and repeated-sprint ability) [3,4,6,7,8,9]. However, some athletes are not easily classified into physical demands that are strictly endurance or strength/power in nature and require multiple facets of health- (e.g., aerobic capacity, muscular strength) and skill-related (e.g., agility, speed, power) physical fitness [10]. Recently, Mielgo-Ayuso addressed this concern within soccer players; however, a majority of the reviewed investigations evaluated aspects of physical performance (i.e., speed, power, agility, time-to-exhaustion) with limited data reported regarding simulated performance [11]. Reasonably, instructing athletes with diverse physical demands to consume caffeine for performance benefits has limited evidence to support its efficacy [11,12]. Since preserving muscle function during competition is important for preventing premature fatigue, investigating the role of acute caffeine supplementation during combined exercise modalities is warranted.

The article "The Effects of Acute Caffeine Supplementation on Performance in Trained CrossFit Athletes" was retracted in 2020. Reasons: errors in the analysis; errors in the methods; errors in the results or conclusions.

In the most recent meta-analysis of the effects of caffeine supplementation on muscle function, the authors reported significant improvements (+6–7%) in muscular endurance after caffeine supplementation [13]. A majority of the 17 investigations cited in the review assessed large muscle group(s) muscular endurance via repetitions to failure over the course of multiple weightlifting sets separated by recovery periods [14,15,16,17]. These investigations utilized isotonic exercise machines and reported relatively low repetitions (<30) even over the course of multiple sets, which may not fully translate to athletic performance.

The recent dramatic increase in high-intensity functional training—which aims to enhance multiple domains of physical fitness by temporally exposing athletes to varying modes of exercise (e.g., endurance, resistance) within and between each session, for varying durations (e.g., 2–60 min), at a relatively high-intensity [18]—has been primarily driven by CrossFit which has an annual competition called the CrossFit Games [18,19,20,21,22]. Within the athletic performance environment of CrossFit, repetitions can approach up to 700 in a 20-min training session [21,23]. Similar to other sports, CrossFit athletes likely possess high-levels of health- and skill-related aspects of physical fitness and research has significantly correlated CrossFit performance with aerobic capacity, muscular strength (upper- and lower-body), and power [20,23,24]. Unfortunately, limited evidence from the sports nutrition community exists regarding the utility of dietary supplementation for CrossFit performance [25].

To the best of our knowledge, no investigations have examined the effect of caffeine supplementation on CrossFit performance. Ostensibly, caffeine represents an ideal candidate for investigation with ‘good evidence’ establishing its ergogenicity across a variety of exercise protocols (e.g., endurance, high-intensity, muscular endurance, sprint performance, maximal strength) and muscle groups [3,26,27]. However, the effects of caffeine supplementation on performance during a high-volume muscular endurance workouts that tax multiple muscle groups with limited recovery remains unknown. In this study, we examined the effects of caffeine supplementation on CrossFit performance for a 20-min muscular endurance workout (‘Cindy’). Similar to previous investigations documenting caffeine’s ergogenic effects for other types of training programs [3,26,27], we hypothesized that caffeine supplementation would result in an increase in CrossFit performance during a high-volume muscular endurance workout which taxed multiple muscle groups with limited recovery as well as a decrease in perceptual responses to exercise (i.e., perceived exertion). 

The article "The Effects of Acute Caffeine Supplementation on Performance in Trained CrossFit Athletes" was retracted in 2020. Reasons: errors in the analysis; errors in the methods; errors in the results or conclusions.

## 2. Materials and Methods

### 2.1. Design and Participants

This study used a randomized, double-blind, crossover design to determine the effects of caffeine on CrossFit performance. Inclusion criteria were: ≥6 months of CrossFit experience; previously completing ‘Cindy’ or a workout with similar repetition volumes for the included movements; male sex; and 18–45 years of age. Participants were excluded if they had any known health-problem (e.g., physical and mental), answered ‘Yes’ to any physical activity readiness questionnaire items, reported allergic or negative side-effects with caffeine use, were unable to perform ‘Cindy’ as prescribed, or were taking medication for seizures. This research project was approved by Kansas State University’s Institutional Review Board (#9100). All subjects completed a brief online survey to determine eligibility and provided written informed consent for the study in person.

### 2.2. Measures and Procedures

Participants were asked to refrain from caffeine, alcohol, vigorous exercise, and nicotine for 24 h, maintain their normal diet, adequately hydrate, refrain from eating 3 h prior to testing, and to otherwise maintain their usual training regimen throughout the study. Anthropometric measures were taken on the first laboratory visit. Height was measured using a stadiometer. Body mass and percent body fat were determined using a bioelectrical impedance analysis in standard mode (TBF-300A; Tanita, Japan). Following anthropometric measures, participants (n = 13, age = 28.5 ± 6.6 years; height = 178.9 ± 5.1 cm; mass = 84.3 ± 9.9 kg; percent body fat = 20.1 ± 2.9%; experience = 49.2 ± 36.3 months) were randomized to consume either caffeine or the placebo. To determine treatment order (placebo then caffeine vs. caffeine then placebo), participants were randomized using a random number generator (0–99) with odd numbers being placed into the placebo condition and even numbers being placed into the caffeine condition for the first visit (placebo then caffeine: n = 7; caffeine then placebo: n = 6). The caffeine pill(s) (Prolab) were provided at 5 mg·kg^−1^ body mass [28]. A 300 μg biotin pill(s) was used as a placebo to match for color and texture of caffeine pills. The same amount of pill(s) of biotin were administered as caffeine pills to ensure blinding. Participants began a self-selected warm-up 50-min after consumption of the pill(s). Participants began the CrossFit workout—‘Cindy’—60-min after consumption of the pill(s). The workout was performed indoors in a gym with the temperature set to 22 °C. Each participant performed the workout alone with no clock or timing device visible to them and without music. ‘Cindy’ was chosen since it is a standardized CrossFit workout, and it has been previously described in the literature [21,22,29]. Briefly, participants completed as many rounds as possible of 5 pull-ups, 10 push-ups, and 15 air squats in 20 min. CrossFit movement standards were followed; kipping was allowed for the pull-ups; push-ups were performed on the toes, with the subject lowering himself with a straight body until his chest touched the floor; and air squats required subjects to reach full knee and hip extension at the top of each repetition and have their hip crease below their knee at the bottom of each repetition [29]. Judges, with CrossFit Level 1 or 2 Certificates, verbally counted repetitions. Repetitions that did not meet movement standards were not counted, and participants were provided feedback to meet the movement standards. CrossFit performance was the total number of repetitions completed in 20 min. Participants were given a post-exercise survey to determine their rate of perceived exertion (RPE) achieved during the workout on a scale of 1–10 [30]. Participants returned to the laboratory after a 7-day washout period, consumed the opposite pill(s) from their first visit (placebo n = 6; caffeine n = 7), and identical procedures were followed for the workout and post-workout survey. For each participant, the testing sessions were scheduled within a 2 h window. Percent change in the performance (i.e., repetitions completed) was calculated to assess the individual effects of caffeine supplementation [(caffeine − placebo)/(placebo) × 100)]. Individuals were classified as ‘non-responders’ if the percent change was <1%.

The article "The Effects of Acute Caffeine Supplementation on Performance in Trained CrossFit Athletes" was retracted in 2020. Reasons: errors in the analysis; errors in the methods; errors in the results or conclusions.

### 2.3. Analysis

Data were entered into SPSS 25 (Armonk, NY, USA) for analysis. Dependent variables were tested for normality using the Kolmogorov-Smirnov test. The variables were normally distributed and were described as mean and standard deviation. Paired samples t-tests were used to determine differences between the caffeine and placebo conditions in the total number of repetitions and RPE. An additional paired samples t-test was used to determine if a learning effect was present between the first and second sessions. An analysis of covariance was used to determine differences in the total number of repetitions performed during the caffeine condition between treatment order groups (placebo-caffeine vs. caffeine-placebo) while controlling for the total number of repetitions performed during the placebo condition. Descriptive data are provided as mean ± standard deviation. Degrees of freedom (df), critical value (cv), level of significance (p), and effect size (ES) were reported for each paired samples t-test (t). The magnitude to treatment effects (ES) were estimated with Cohen’s D and classified as “trivial” (<0.19), “small” (0.20–0.49), “moderate” (0.50–0.79), and “large” (>0.80) [31]. A significance level was set at *p* < 0.05.

## 3. Results

Participants significantly improved CrossFit performance (i.e., total number of repetitions performed) during the caffeine trial (461.4 ± 103 repetitions) as compared to placebo (425.0 ± 93.5 repetitions), *t*(12) = −3.928, *p* = 0.002, ES = 0.39 (Figure 1). No significant differences were found for perceptual exercise responses (i.e., RPE) between the caffeine (8.5 ± 1.3) and the placebo conditions (8.3 ± 1.3), *t*(12) = −0.562, *p* = 0.584 (Figure 2). No significant learning effect was identified between the first and second sessions (445.6 ± 95.0 vs. 440.8 ± 105.0 repetitions, *t*(12) = 0.348, *p* = 0.73). After controlling for the total number of repetitions performed during the placebo condition, no significant treatment order effect was observed for the total number of repetitions performed during the caffeine condition between treatment order groups (F(1,13) = 0.760, *p* = 0.40). Figure 3 shows the percent change in performance (i.e., total repetitions) [(caffeine − placebo)/(placebo) × 100)] performed across all subjects (8.9%, 95% CI (4.0–13.7%)), three of whom were ‘non-responders’ (−0.5%, −0.4%, 0.27%).

## 4. Discussion

The purpose of our investigation was to determine the effects of acute caffeine supplementation on CrossFit performance and perceptual responses to exercise in CrossFit-trained males. Because of the well-documented ergogenic effects of caffeine that are likely due to central mechanisms [2,3,4,5], we hypothesized that caffeine supplementation would improve CrossFit performance. Our hypothesis was partially supported with significant improvements in CrossFit performance with no changes in perceptual responses after caffeine supplementation. Additionally, we tested for a learning effect between the first and second session of ‘Cindy’ and found no significant differences. Lastly, our study aimed to provide a novel contribution to the literature regarding caffeine supplementation and muscular endurance by providing a unique high-volume muscular endurance challenge. On average, participants in the current investigation performed over 400 repetitions for the 20 min workout during the caffeine and placebo conditions, which we believe adequately addressed this challenge. To the best of our knowledge, this is the first study to determine the effects of caffeine supplementation on performance during any CrossFit workout, which taxed multiple muscle groups for an extended period of time with minimal rest.

The article "The Effects of Acute Caffeine Supplementation on Performance in Trained CrossFit Athletes" was retracted in 2020. Reasons: errors in the analysis; errors in the methods; errors in the results or conclusions.

In the current study, caffeine supplementation (5 mg·kg^−1^ body mass) increased mean CrossFit performance by 8.9%. Caffeine’s ergogenic effect has been reported to improve performance by 5.5–8.5% during other repeated-high-intensity efforts in team sports athletes, and by 6–7% during muscular endurance exercise [6,13,32]. Previous investigations determining the effects of caffeine supplementation on muscular endurance had participants perform a comparatively low number of repetitions (<30) until failure over numerous sets (≥3), separated by rest periods, and were usually within isolated muscle groups [16,17,33]. Our investigation provides a unique addition to the literature as our participants were instructed to complete as much work as possible within the 20-min time limit while utilizing multiple multi-joint body weight exercises. Multi-joint exercises have been speculated to increase RPE [3]; however, similar to some investigations, we failed to detect statistically significant changes in RPE between the caffeine and placebo conditions [16,33,34]. However, other investigations assessing the effects of caffeine on RPE during resistance training exercise have provided mixed results [3]. Thus, researchers might consider additional measurements of during-workout exertion since RPE is usually taken after the exercise bout given the nature of resistance exercise [35].

Our study assessed CrossFit performance via ‘Cindy’, which has been the most studied CrossFit workout to date [21,22,29]. Butcher and colleagues reported ‘Cindy’ performance between competitive, experienced, and novice CrossFit athletes completing 698, 469, 389 repetitions, respectively [21,23]. The current study, which aimed to recruit CrossFit-trained (i.e., experienced) participants, seems to follow those trends. Moreover, Crawford [24] measured work capacity derived from performance during a similar CrossFit workout and reported ~16% increase in work capacity after 6 weeks of a high-intensity functional training intervention which followed a CrossFit template for novice healthy adult participants. This is promising for researchers and practitioners alike as the use of benchmark workouts, such as ‘Cindy’, may be sensitive enough to detect changes in CrossFit performance from ergogenic aids (e.g., exercise training interventions, nutrient modification) [21].

The article "The Effects of Acute Caffeine Supplementation on Performance in Trained CrossFit Athletes" was retracted in 2020. Reasons: errors in the analysis; errors in the methods; errors in the results or conclusions.

Strengths of the current investigation include a robust study design with subjects serving as their own controls, the recruitment of trained male CrossFit participants who were able to complete ‘Cindy’ as prescribed as a high-volume muscular endurance workout, and it is the first study to document an ergogenic effect during a CrossFit workout. However, our study does not go without limitation. Although 13 CrossFit-trained men completed our study, our sample size is reasonably small. However, the average sample size reported in a recently published systematic review on the effects of caffeine in trained soccer players was 15 participants; therefore, our investigation reflects similar sample sizes compared to other studies regarding caffeine’s ergogenic effect in trained populations [11]. Participant training volume was not reported leading up or during the investigation. Although participants were instructed not to exercise vigorously for 24 h prior to each testing session or change their training regimen during the study period, fatigue and/or delayed onset muscle soreness from other training sessions could impact our results. Additionally, our study lacked more invasive measures to determine blood caffeine concentration and caffeine metabolism. Recently identified, caffeine supplementation may have a ‘responder’ vs. ‘non-responder’ nature, which limits the translation of our investigation to ‘non-responder’ populations [27]. In our investigation, we had three participants (−0.5%, −0.4%, 0.27%) who were ‘non-responders’ to caffeine supplementation (Figure 2). The inter-individual differences in the ergogenicity of caffeine are thought to be related to genetic polymorphisms associated with the CYP1A2 and ADORA2A genes, which discern fast and slow caffeine metabolism/clearance [36]. Although the current investigation did not characterize the genetic differences among our participants, these differences may explain the ‘responder’ vs. ‘non-responder’ nature of our findings and present an avenue for future investigations. However, to truly elucidate ‘responders’ vs. ‘non-responders’, a baseline control condition where no supplements are provided to the participants prior to the exercise bout is necessary. Additionally, our study investigated the effects of caffeine supplementation on CrossFit performance for males and may not be generalizable to female participants. Caffeine supplementation in females is complicated by the effects of estrogen and oral contraceptive steroids on caffeine metabolism, both of which appear to prolong the effects of caffeine in the body [3,37]. To increase internal validity, participants performed the workout alone, with no clock visible, and no music was playing. Results may differ when ‘Cindy’ is performed in a group setting with a visible clock and music playing [38,39,40]. Lastly, our investigation utilized a 10-point Likert scale for RPE and may not be sensitive enough to capture perceptual changes during CrossFit protocols. Although mixed results exist for 10-point and 15-point scales for RPE during caffeine supplementation utilizing resistance- and endurance-based protocols, a recent publication by Crawford and colleagues highlight that a 15-point scale may be more appropriate in CrossFit athletes [3,34,35]. 

The article "The Effects of Acute Caffeine Supplementation on Performance in Trained CrossFit Athletes" was retracted in 2020. Reasons: errors in the analysis; errors in the methods; errors in the results or conclusions.

## 5. Conclusions

In conclusion, we have provided evidence that caffeine supplementation at 5 mg·kg^−1^ body mass ingested 60 min prior to the CrossFit workout ‘Cindy’ increased the number of repetitions performed in male CrossFit-trained individuals. However, despite the central effects of caffeine, we found no significant changes in perceptual responses during the exercise bout. Caffeine’s ergogenic effects are well documented in the literature and further supported by our investigation, yet practitioners and athletes should be aware that some ‘non-responders’ may exist; thus, evaluating caffeine’s effectiveness prior to competition for a specific athlete is encouraged.

## Figures and Tables

**Figure 1:** Performance (i.e., repetitions performed) in the caffeine and placebo condition. Data represent mean ± SD. * Significantly different from performance during the placebo condition *p* < 0.05.

**Figure 2:** Perceptual responses to exercise (i.e., ratings of perceived exertion (RPE)) in the caffeine and placebo condition. Data represent mean ± SD.

**Figure 3:** Percent change in performance [(repetitions completed with caffeine − repetitions completed with placebo)/(repetitions completed with placebo) × 100)] in the caffeine and placebo condition for each participant.
